This article has been retracted.

# Soliton dynamics in optical fiber based on nonlinear Schrödinger equation

**DOI:** 10.1016/j.heliyon.2023.e14235

**Published:** 2023-03-08

**Authors:** Harish Abdillah Mardi, Nasaruddin Nasaruddin, Muhammad Ikhwan, Nurmaulidar Nurmaulidar, Marwan Ramli

**Affiliations:** a Mathematics Graduate Program, Faculty of Mathematics and Natural Sciences, Universitas Syiah Kuala, Banda Aceh 23111, Indonesia; b Electrical and Computer Engineering Department, Universitas Syiah Kuala, Banda Aceh 23111, Indonesia; c Department of Mathematics, Faculty of Mathematics and Natural Sciences, Universitas Syiah Kuala, Banda Aceh 23111, Indonesia

**Keywords:** Attenuation, Dispersion, Hamiltonian, NLS equation, Optical fiber

## Abstract

Optical fiber is a component of the green and sustainable internet. This paper analyzes the energy loss induced by the attenuation effect of electromagnetic waves during optical fiber propagation. The dynamics of the Hamiltonian, which was derived using the dynamics of the solution the Nonlinear Schrödinger equation (NLS) problem, were used to investigate the energy drop. In this study, the Newton-Raphson (NR) approach was used to establish the stationary solution of the NLS problem, and the fourth order Runge-Kutta method was used to evaluate the dynamics of the solution (RK4). In this study, numerous parameters are adjusted, including group wave dispersion, nonlinearity, attenuation parameter, and potential trap. The solution of the NR approach is fairly close to the analytical solution based on the analytical solutions. The dynamics of the NLS equation solution are greatly influenced by parameters. The obtained results reveal that for large attenuation parameter values, the strength of the propagating electromagnetic waves decreases quite quickly. The result also shows that the other parameters studied must be maintained at the best conditions to support the attenuation parameters and potential trap. This condition is an indicator in the choice of the fundamental material for producing optical fiber, which should have a low attenuation and dispersion effect.

## 1 Introduction

Research on optical signal processing is an important aspect in optical communication systems because it has a very fast response rate [1]. This is closely related to the use of nonlinear refractive index in optical fiber. If an optical fiber only uses a nonlinear refractive index, then the partial signal can be lost over time. This is due to the non-uniform distribution of intensity in the pulses [2]. Improved system performance can be done by utilizing the natural properties of optical fiber, namely Group Velocity Dispersion (GVD) and Self-Phase Modulation (SPM). The balance of GVD and SPM on an optical fiber can form solitons. Soliton can improve system performance due to its stable propagation along the fiber. The existence of solitons in optical fiber has been observed by experimental observations [3], [4], [5] as well as theoretical studies [6], [7], [8]. Soliton propagation in optical fiber is theoretically approached by an equation which is often called the Nonlinear Schrödinger (NLS) equation [9], [10], [11].

The NLS equation is an equation that can generally be used to observe the dynamics of waves propagating in a nonlinear dispersive medium, such as Bose-Einstein condensation [12], [13], [14], [15], [16], [17], plasma physics [18], [19], [20], double-stranded Deoxyribonucleic Acid (DNA) [21], electric circuit [22], fluid dynamics [23], [24], [25], and many more. In nonlinear optics, the NLS equation can be used to observe the propagation of electromagnetic waves in a single mode optical fiber medium [26], [27]. The NLS equation describes the propagation of electromagnetic waves in the optical fiber which changes slowly [28]. In general, the NLS equation can be written in the form Eq. (1),

(1) $$i\frac{\partial \Psi }{\partial t}+C\nabla^{2}\Psi -V\Psi +F(\Psi )=0,$$

with Ψ≡Ψ(x,t)∈C is a wave function at $t\in R^{+}$, x∈R, *C* is a real value parameter (C∈R). The F(Ψ) term is a nonlinear term that has several forms, including [29]:

**Table:** 

1	Cubic-type nonlinearity	=	|Ψ|^2^Ψ;
2	Quintic-type nonlinearity	=	|Ψ|^4^Ψ;
3	Ablowitz-Ladik type nonlinearity	=	$\frac{1}{2}|\Psi {|}^{2}\frac{\partial \Psi }{\partial x}$.

The uniqueness of the NLS equation makes this equation interesting to study in an effort to develop the NLS equation. This is because for the case of cubic nonlinearity, the NLS equation has an analytical solution, so the NLS equation is classified as an integrable system. Various kinds of nonlinearities in various contexts have been studied from the NLS equation. So that the NLS equation is no longer system integrable. There have been many studies aimed at anticipating this situation. One of the nonlinearities that makes the NLS equation no longer system integrable is the attenuation factor in the NLS equation [30], [31], [32]. The extended simplest equation (ESE) approach, modified Kudryashov (MKud) method, and modified Khater (MKha) method were used to solve the NLS equation using computational computations. The collected findings demonstrate good performance [33]. One example is the Inverse Scattering Transform (IST) which is the only method that can integrate only a few of the nonlinear equations of its time [34]. Transformations between the spacetime domain and the nonlinear spectrum domain underpin IST. The IST spectrum is divided into two parts: a discrete component for solitons and a continuous part for dispersive waves [35]. The IST for decaying data was created, and a single-breathing soliton solution was discovered. The IST equation necessitates different scattering data symmetries than the traditional NLS equation [36]. A spin-like model is gauge equivalent to the nonlocal complex modified Korteweg-de Vries (mKdV) equation [37]. The gauge equivalence shows that the nonlocal complex mKdV equation and the classical complex mKdV equation have a considerable difference. The Darboux transformation (DT) for the nonlocal complex mKdV equation is used to produce a number of exact solutions, including dark soliton, W-type soliton, M-type soliton, and periodic solutions. The soliton solution is also obtained using the Jacobian-elliptic-function (JEF), especially in the high-order NLS [38]. JEF produces seed solutions or ansatz, while DT uses the linearly-independent and non-periodic solutions to obtain soliton solutions. A variety of soliton solutions can also be found in NLS using the concept of the Laplacian operator in fractal dimensions and the concept of ansatz variety [39], [40]. With the NLS envelope of the KdV waveform, the NLS equation has various nonlinear and dispersion coefficients [25].

Attenuation in nonlinear optics is wave attenuation that occurs when electromagnetic waves interact with the medium [41], [42], [43], [44]. Due to the attenuation effect on the optical fiber, electromagnetic waves lose energy as they propagate in the optical fiber [45], [46], [47]. This article attempts to present the limitations and advantages of a medium in optical fiber based on attenuation as shown in the NLS equation solution. This study discusses the Hamiltonian distribution using the NLS equation in an effort to analyze the energy of electromagnetic waves in optical fiber with variations in the attenuation effect. The solution of the NLS equation is determined using the Newton-Raphson (NR) method [48], [49], [50], [51] and the dynamics of the solution will be analyzed using the fourth order Runge-Kutta method (RK4) [52], [53], [54]. The systematic writing of this report consists of section 2, section 3, and section 4. Section 2 focuses on NLS equations, starting from analytical and numerical solutions to NLS equations and the methods used. Section 3 presents the results and discussion of this research, which consists of simulating the solution of the NLS equation and the dynamics of the solution to the NLS equation in an effort to analyze the energy attenuation that occurs in the dynamics of the solution by obtaining a Hamiltonian distribution. In section 4, the conclusions obtained in this study will be described. This study has been carried out in Laboratory of Applied Mathematics Syiah Kuala University in 2022.

## 2 Nonlinear Schrödinger equation

The NLS equation is a second-order nonlinear partial differential equation that can explain the dynamics of wave propagation in a nonlinear dispersive medium. The NLS equation that will be used in this study can be written in the form of,

(2) $$i\frac{\partial \Psi }{\partial t}+\frac{\beta }{2}\frac{\partial^{2}\Psi }{\partial x^{2}}+\gamma |\Psi {|}^{2}\Psi =V(x)\Psi -i\frac{\alpha }{2}\Psi ,$$

with Ψ(x,t) is the complex envelope of the electric field that propagates in the optical fiber, *β* is the group wave dispersion parameter, *γ* is the third-order nonlinearity, V(x) is the trapping potential, the *α* parameter represents the attenuation in the optical fiber, and *x* and *t* respectively represent dimensionless spatial and time variables. From Eq. (2), we can derive the normalized equation of motion (*Q*) and its Hamiltonian (*H*) which can be written as,

$$Q=\int_{-\infty }^{\infty }|\Psi {|}^{2}dx,H=\frac{1}{2}\int_{-\infty }^{\infty }\left[\frac{\beta }{2}{\left(\frac{d\Psi }{dx}\right)}^{2}+\frac{\gamma }{2}|\Psi {|}^{4}-V(x)|\Psi {|}^{2}+i\frac{\alpha }{2}|\Psi {|}^{2}\right]dx.$$

Hamiltonian is explained by deriving from basic physical laws, such as norms and the conservation of energy. The law of conservative energy leads to vertex conditions and generalized Kirchhoff's rules [55], [56]. The Hamiltonian represented in the conservative energy form is conserved due to the loss of its attenuation effect. In contrast to the use of the PDE system, which produces a different Hamiltonian [57]. This article incorporates attenuation parameters and potential devices in its Hamiltonian calculations. As a result, the calculation of H in this paper needs to go through calculations that have the same principles as those done in previous studies [58].

### 2.1 Analitical solution of the nonlinear Schrödinger equation

The analytical solution of the NLS equation can be constructed if the two parameters in Eq. (2), namely V(x) and *α* is zero (V(x)=α=0). Hence, Eq. (2) can be written as,

(3) $$i\frac{\partial \Psi }{\partial t}+\frac{\beta }{2}\frac{\partial^{2}\Psi }{\partial x^{2}}+\gamma |\Psi {|}^{2}\Psi =0.$$

The solution to Eq. (3) can be constructed by substituting ansatz in the form,

(4) $$\Psi (x,t)=\psi (x)e^{i\Omega t},$$

where Ω is a real value parameter (Ω∈R). By substituting Eq. (4) into Eq. (3), we get an analytical solution to the NLS equation which can be written as,

(5) $$\Psi (x,t)=\sqrt{\frac{2\Omega }{\gamma }}sech\left(\sqrt{\frac{2\Omega }{\beta }}x\right)e^{i\Omega t}.$$

### 2.2 Numerical solution of the nonlinear Schrödinger equation

Eq. (2) is a non-integrable system, which can be interpreted as having no analytical solution. Many semi-analytic and numerical methods are offered to find the solution of Eq. (2), including the sine-cosine method, the IST method, the tanh-coth method, the Darboux transformation method, the F expansion method, the Hirota bilinear method, the Bäcklund and Auto-Bäcklund transformation method, modified Khater method, exponential cubic B-spline differential quadrature method and many more [33], [37], [59], [60], [61], [62]. This research will use a numerical method known as Newton-Raphson (NR) method to find a stationary solution numerically to the NLS equation. The ansatz NLS equation written in Eq. (4) is substituted into Eq. (2) and the resulting equation is of the form,

(6) $$-\Lambda \psi +\frac{\beta }{2}\frac{d^{2}\psi }{dx^{2}}+\gamma \psi^{3}=V(x)\psi -i\frac{\alpha }{2}\psi .$$

Eq. (6) can be transformed into a function which can be written as,

(7) $$f(\psi )=-\Lambda \psi_{n}+\frac{\beta }{2}\frac{d^{2}\psi_{n}}{dx^{2}}+\gamma \psi_{n}^{3}-V(x)\psi_{n}+i\frac{\alpha }{2}\psi_{n}=0,\psi \in R,\;n=-N,-N+1,\ldots ,N-1,N,\;N\in Z^{+}.$$

The NR method can be applied to find a solution to Eq. (7) with the form,(8) where Eq. (8) used variable Eq. (9), Eq. (10), and Jacobian matrix Eq. (11)(9)

(10) $$\frac{d\psi }{dx}=\frac{1}{2\pi }\int_{-\infty }^{\infty }ikdk\int_{-\infty }^{\infty }d\xi e^{ik(x-\xi )}\psi (\xi ),$$

(11) $$J=[\begin{array}{cccccc} i\Omega +3i\gamma \psi_{-N}^{2}-iV(x)-\frac{\alpha }{2} & i\frac{\beta }{2} & \ldots & \ldots & \ldots & \ldots \\ i\frac{\beta }{2} & \ddots & \ddots & \ldots & \vdots & \vdots \\ \vdots & \ddots & \ddots & \ddots & \vdots & \vdots \\ \vdots & \vdots & \ddots & \ddots & \ddots & \vdots \\ 0 & \ldots & \ldots & i\frac{\beta }{2} & i\Omega +3i\gamma \psi_{0}^{2}-iV(x)-\frac{\alpha }{2} & i\frac{\beta }{2}\\ \vdots & \vdots & \vdots & \vdots & \ddots & \ddots \\ \vdots & \vdots & \vdots & \vdots & \vdots & \ddots \\ \vdots & \vdots & \vdots & \vdots & \vdots & \vdots \\ 0 & \ldots & \ldots & \ldots & \ldots & \ldots \end{array}$$

The solution to the NLS equation using the NR method will be determined using an initial guess in the form,

(12) $$\psi_{0}=\sqrt{2}sech(\sqrt{2}x).$$

Eq. (12) is selected based on the analytical solution of the NLS equation that has been written in Eq. (5).

### 2.3 Runge-Kutta 4${}^{th}$ order

The RK4 method can be applied to the NLS equation by transforming the NLS equation into the form,

(13) $$y_{i+1}=y_{i}+hf(x_{i},y_{i}),$$

by using ODE in Eq. (13), then the RK4 method can be applied by using Eq. (14) [63],

(14) $$k_{1}=hf(x_{i},y_{i}),k_{2}=hf(x_{i}+\frac{h}{2},y_{i}+\frac{k_{1}}{2}),k_{3}=hf(x_{i}+\frac{h}{2},y_{i}+\frac{k_{2}}{2}),k_{4}=hf(x_{i}+h,y_{i}+k_{3}),y_{i+1}=y_{i}+\frac{1}{6}(k_{1}+2k_{2}+2k_{3}+k_{4}).$$

## 3 Result and discussion

The Hamiltonian dynamics in this study were constructed using the dynamics of the solution to the NLS equation using the RK4 method. Before getting the dynamics of the solution of the NLS equation, it is necessary to find a stationary solution of the NLS equation using the NR method. The stationary solution of the NLS equation is used as an input signal which is then entered in the RK4 method which represents the propagation of electromagnetic waves in the optical fiber. The Hamiltonian obtained in this study represents the energy of electromagnetic waves propagating in the optical fiber. Meanwhile, the Hamiltonian dynamics obtained in this study were analyzed in order to pay attention to the effect of the various parameters on the energy of electromagnetic waves propagating in the optical fiber. The parameter values that are varied in the study are dimensionless, so that each result listed in this paper does not have units.

### 3.1 Solution of the nonlinear Schrödinger equation without potential traps

The solution to the NLS equation without a trap potential (V(x)=0) with variations in the value of *β* and parameter *γ* which has a fixed value has been simulated as shown in Fig. 1.

**Figure 1:** Solution of the NLS equation with *V*(*x*)=0 and *γ* = 1 for (a) *β* = 1, (b) *β* = 1.7, and (c) *β* = 2.5.

Fig. 1 represents a simulation of the solution of the NLS equation for the parameter value β∈[1,2.5]. Based on Fig. 1, it is found that the widening that occurs in the electromagnetic wave pulse is associated with an increase in the value of parameter *β*. The greater the value of *β*, the wider the pulse of electromagnetic waves entering the optical fiber. This difference is indicated by observing Fig. 1(a) with β=1 having a narrow pulse when compared to Fig. 1(b) and Fig. 1(c) with β=1.7 and β=2.5, respectively.

Fig. 2 represents a simulation of the solution of the NLS equation for the parameter value γ∈[1,2.5]. Based on Fig. 2, it is found that parameter *γ* affects the amplitude of the electromagnetic wave without affecting the pulse width of the wave. This is indicated by observing Fig. 2(a) where γ=1 has the highest amplitude when compared to Fig. 2(b) and Fig. 2(c).

**Figure 2:** Solution of the NLS equation with *V*(*x*)=0 and *β* = 1 for (a) *γ* = 1, (b) *γ* = 1.7, and (c) *γ* = 2.5.

Changes in *β* and *γ* values are more precisely displayed in two dimensions in this simulation, demonstrating that the *β* parameter magnifies the pulse and the *γ* parameter is connected to amplitude.

### 3.2 Solution of the nonlinear Schrödinger equation with potential traps

The solution of the NLS equation in the presence of a trap potential $\left(V(x)=\frac{1}{2}x^{2}\right)$ with a variable value of *β* and a constant value of parameter *γ* has been simulated as shown in Fig. 3.

**Figure 3:** Solution of the NLS equation with $V(x)=\frac{1}{2}x^{2}$ and *γ* = 1 for (a) *β* = 1, (b) *β* = 1.7, and (c) *β* = 2.5.

Fig. 3 represents a simulation of the solution of the NLS equation for the parameter value β∈[1,2.5]. As shown in Fig. 3, it can be seen that the variation of *β* affects the amplitude and pulse width of the electromagnetic wave in the optical fiber. It can be seen in Fig. 3(a) that β=1 has a shorter amplitude and narrower pulse than the solution of the NLS equation shown in Fig. 3(b) for β=1.7 and Fig. 3(c) for β=2.5. After getting a simulation of the solution of the NLS equation with potential traps for the case of variation *β*, the solution of the NLS equation with varying values of parameter *γ* and parameter *β* which has a fixed value has been shown in Fig. 4.

**Figure 4:** Solution of the NLS equation with $V(x)=\frac{1}{2}x^{2}$ and *β* = 1 for (a) *γ* = 1, (b) *γ* = 1.7, and (c) *γ* = 2.5.

Fig. 4 represents a simulation of the solution of the NLS equation for the parameter value γ∈[1,2.5]. As shown in Fig. 4, it can be seen that the variation of *γ* affects the amplitude height without affecting the pulse width of the electromagnetic wave in the optical fiber. It can be seen in Fig. 4(a) that γ=1 has a higher amplitude than the solution of the NLS equation shown in Fig. 4(b) for γ=1.7 and Fig. 4(c) for γ=2.5.

### 3.3 Dynamics of the nonlinear Schrödinger equation

We numerically study the dynamics of solitons in the NLS equation with several values of *α*, *β*, and *γ* for the case V(x)=0 and $V(x)=\frac{1}{2}x^{2}$ in order to analyze the attenuation effect that occurs when electromagnetic waves interact with optical fiber. The dynamics of the solution of the NLS equation with V(x)=0 and γ=1 for the case of several values of *α* and *β* are obtained as shown in Fig. 5.

**Figure 5:** Dynamics of the solution of the NLS equation with *V*(*x*)=0, *γ* = 1 and *β* = 1 (top), *β* = 1.7 (middle), and *β* = 2.5 (bottom) for *α* = 0.01 (left), *α* = 0.05 (center), and *α* = 0.1 (rigth).

Fig. 5 represents the dynamics of the solution of the NLS equation with V(x)=0 and γ=1 for the case of several values of *α* and *β*. Based on the results that have been illustrated in Fig. 5, it was found that the values of *β* and *α* greatly affect the condition of the electromagnetic waves that propagate in the optical fiber. The effect of parameter *β* with a relatively large value on electromagnetic waves causes the electromagnetic wave pulses that propagate in the optical fiber to widen. Meanwhile, parameter *α* is very influential on the height of the electromagnetic wave amplitude with its relation to the intensity of the electromagnetic wave. The greater the value of *α*, the faster the electromagnetic wave loses its intensity. After getting the results of the dynamics of the solutions of the NLS equations for variations *α* and *β*, the dynamics of the solutions of the NLS equations for variations in the values of *α* and *γ* are simulated as shown in Fig. 6.

**Figure 6:** Dynamics of the solution of the NLS equation with *V*(*x*)=0, *β* = 1 and *γ* = 1 (top), *γ* = 1.7 (middle), and *γ* = 2.5 (bottom) for *α* = 0.01 (left), *α* = 0.05 (center), and *α* = 0.1 (rigth).

Fig. 6 represents the dynamics of the solution of the NLS equation with V(x)=0 and β=1 for the case of several values of *α* dan *γ*. Based on Fig. 6, it can be seen that for each variation of *γ* only affects the amplitude of the electromagnetic wave when it enters the optical fiber. The dynamics of the solution of the NLS equation simulated in Fig. 6 show the same shape and decrease in amplitude, only the magnitude of the amplitude is different. The relatively large value of the *γ* parameter causes a decrease in the amplitude of the electromagnetic wave at the beginning of propagation.

The dynamics of the solution of the NLS equation for the case of $V(x)=\frac{1}{2}x^{2}$ is also presented in this study with several values of *α*, *β*, and *γ*. The dynamics of the solution of the NLS equation for the case of $V(x)=\frac{1}{2}x^{2}$ and γ=1 and some values of *α* and *β* are obtained as illustrated in Fig. 7.

**Figure 7:** Dynamics of the solution of the NLS equation with $V(x)=\frac{1}{2}x^{2}$, *γ* = 1 and *β* = 1 (top), *β* = 1.7 (middle), and *β* = 2.5 (bottom) for *α* = 0.01 (left), *α* = 0.05 (center), and *α* = 0.1 (rigth).

Fig. 7 represents the dynamics of the solution of the NLS equation with $V(x)=\frac{1}{2}x^{2}$ and γ=1 for the case of several values of *α* and *β*. As has been simulated in Fig. 7, it can be observed that the trapping potential in the optical fiber can reduce the spread of waves that occur during the propagation of electromagnetic waves. This can be analyzed from the dynamic form of the solution of the NLS equation which is only right in the middle of the optical fiber for every time and every value of *β* without spreading in all directions as shown in Fig. 7. Because there is no propagation of electromagnetic waves in the fiber, the intensity of electromagnetic waves propagating in the optical fiber in the presence of a trapping potential is reduced in a relatively longer period of time compared to Fig. 5. Thus, indirectly the presence of trapping potential in the optical fiber can reduce the effects of dispersion and attenuation experienced by electromagnetic waves when propagating in the optical fiber. The dynamics of the solution of the NLS equation for variations in the values of *α* and *γ* have also been simulated as shown in Fig. 8.

**Figure 8:** Dynamics of the solution of the NLS equation with $V(x)=\frac{1}{2}x^{2}$, *β* = 1 and *γ* = 1 (top), *γ* = 1.7 (middle), and *γ* = 2.5 (bottom) for *α* = 0.01 (left), *α* = 0.05 (center), and *α* = 0.1 (rigth).

Fig. 8 represents the dynamics of the solution of the NLS equation with $V(x)=\frac{1}{2}x^{2}$ and β=1 for the case of several values of *α* and *γ*. As shown in Fig. 6 and Fig. 7, the variation in the value of *γ* only causes a decrease in the amplitude at the beginning of the electromagnetic wave. However, the decrease in the intensity of electromagnetic waves that occur when propagating in an optical fiber requires the same time span for each value of *γ*.

### 3.4 Hamiltonian dynamics of the nonlinear Schrödinger equation

The dynamics of the Hamiltonian NLS equation are analyzed in this study to analyze the energy of electromagnetic waves in the optical fiber with attenuation and dispersion effects. The dynamics of the Hamiltonian for the case without trap potential (V(x)=0) and several values of *α*, *β*, and *γ* are obtained as shown in Fig. 9.

**Figure 9:** Dynamics of Hamiltonian NLS equations with *V*(*x*)=0, for *α* = 0.01, *α* = 0.05, and *α* = 0.1 with (a) *β* = 1 and *γ* = 1, (b) *β* = 1.7 (top) and *β* = 2.5 (bottom) for *γ* = 1, and (c) *γ* = 1.7 (top) and *γ* = 2.5 (bottom) for *β* = 1.

Fig. 9 showed the dynamics of Hamiltonian NLS equations with V(x)=0 with several values of *α*, *β*, and *γ*. The Hamiltonian dynamics shown in Fig. 9 illustrates the energy of electromagnetic waves propagating in an optical fiber with several parameter values *α*, *β*, and *γ*. As can be analyzed through Fig. 9, it can be seen that there is a decrease in the energy of electromagnetic waves when propagating in an optical fiber with several values of *α*. The influence of parameter *β* in Fig. 9(a) and Fig. 9(b) on electromagnetic waves causes an increase in energy at t=0. This indicates that the greater the value of parameter *β* indirectly causes the electromagnetic waves propagating in the fiber to increase in energy, but the decrease in energy also increases with time. Meanwhile, parameter *γ* in Fig. 9(a) and Fig. 9(c) causes a decrease in energy at t=0. Thus, the electromagnetic waves propagating in the optical fiber with a large *γ* parameter value causes its energy to decrease slowly. Parameter *α* causes a decrease in energy that occurs along the propagation of electromagnetic waves. The tendency of a high value of *α* causes electromagnetic waves to lose energy so that the amplitude decreases during propagation. The decrease in energy that occurs is caused by various factors, including the effects of attenuation, dispersion, and the interaction of waves with the medium during propagation. This indicates that it is necessary to review the selection of the basic material for making optical fiber to maximize the propagation of electromagnetic waves.

The second case in Hamiltonian dynamics is that the trap potential $V(x)=\frac{1}{2}x^{2}$ in the optical fiber has been simulated as shown in Fig. 10. Fig. 10 represents the dynamics of the Hamiltonian in the NLS equation for the case of $V(x)=\frac{1}{2}x^{2}$ with several values of *α*, *β*, and *γ*. From the figure, it can be analyzed that there is a fluctuation in the energy of the electromagnetic wave that propagates in the optical fiber in the presence of a trap potential and an increase in the energy of the electromagnetic wave. Each parameter that is varied in this case has the same effect as for the case without potential traps. The greater the value of the parameter *β* (see Fig. 10(a) and Fig. 10(b)) causes the energy of the electromagnetic waves propagating in the optical fiber to increase at t=0, but the decrease in energy is also getting faster as it progresses. The greater the value of the *γ* (see Fig. 10(a) and Fig. 10(c)) parameter causes a decrease in energy at t=0, and over time it decreases slowly. A high value of parameter *α* causes electromagnetic waves to lose energy so that the amplitude decreases during propagation. The amplitude of the NLS equation is closely related to the intensity of the electromagnetic wave propagating in the optical fiber. When compared to the simulation results obtained in Fig. 9 and Fig. 10, the use of optical fiber with potential traps in it has a higher efficiency level. This is indicated by the energy of electromagnetic waves propagating in the optical fiber in the presence of a higher trapping potential than the energy of electromagnetic waves propagating in the optical fiber without a trapping potential.

**Figure 10:** Dynamics of Hamiltonian NLS equations with $V(x)=\frac{1}{2}x^{2}$, for *α* = 0.01, *α* = 0.05, and *α* = 0.1 with (a) *β* = 1 and *γ* = 1, (b) *β* = 1.7 (top) and *β* = 2.5 (bottom) for *γ* = 1, and (c) *γ* = 1.7 (top) and *γ* = 2.5 (bottom) for *β* = 1.

The results obtained show that for large attenuation parameter values, the decrease in the intensity of the electromagnetic waves that propagate occurs very quickly. This is an indicator in the selection of the basic material for making optical fiber, which is recommended to have a fairly small attenuation and dispersion effect. The obtained Hamiltonian dynamics decreased during propagation. This indicates that the attenuation effect causes electromagnetic waves to not be able to maintain their energy as they propagate. With the trap potential, the dynamics of the Hamiltonian of the NLS equation represents the energy of the electromagnetic wave which increases at the beginning of propagation and fluctuates during propagation. The effect of the attenuation parameters and the trapping potential on the nonlinear part makes the wave distance longer. However, based on the explanation of the beta and gamma parameters, the influence of these two variables will affect the intensity and diversity of the waves at the source. This means that these four parameters must be maintained in their best condition on a particular medium. This is an indicator that the use of potential traps in optical fiber has a higher efficiency than optical fiber that does not use potential traps. Based on the results obtained, the use of the main material for making optical fiber cores needs to be further reviewed on the effects of attenuation, dispersion, and nonlinearity of materials in order to obtain maximum electromagnetic wave propagation.

## 4 Conclusions

A study has been conducted on the dynamics of the solution to the NLS equation and its Hamiltonian dynamics. First of all, we search for solutions to the NLS equation using the NR method. Based on the results obtained, it appears that the NR method used in this study produces a solution that is very close to the analytical solution of the NLS equation. In the case without potential traps, parameter *β* only affects the pulse width of the electromagnetic wave that is the input signal. Meanwhile, parameter *γ* only affects the high amplitude of electromagnetic waves. In the case of a potential trap, parameter *β* affects the pulse width and increases the amplitude of the electromagnetic wave that becomes the input signal. Meanwhile, parameter *γ* has the same effect as the case without potential traps.

The dynamics of the solution of the NLS equation has been studied in this study numerically using the RK4 method. The dynamics of the solution of the NLS equation is carried out by inputting a signal in the form of a stationary solution of the NLS equation determined using the NR method. Based on the results obtained, in the case without trapping potential, it was found that the dynamics of the solution to the NLS equation which represents the propagation of electromagnetic waves in the optical fiber are dispersed and experience a decrease in intensity for large values of *α* and *β* Whereas in the case without trapping potential, the dynamics of the solution of the simulated NLS equation shows that the intensity decreases but the trapping potential can minimize the dispersion effect on the optical fiber. This is obtained by observing that the electromagnetic waves that propagate in the optical fiber do not experience pulse widening and do not experience wave propagation. Thus, the use of optical fiber with a potential trap is highly recommended when compared to optical fiber without a potential trap.

The dynamics of the Hamiltonian NLS equation have been studied in this study numerically by taking into account each energy during the propagation of electromagnetic waves in the optical fiber. Interesting things arise in the case of potential pitfalls. In the case of a potential trap, the dynamics of the Hamiltonian fluctuates. This is not the case in the case without potential traps. The attenuation effect in optical fiber causes the wave energy to decrease over time. Further studies need to be carried out in this area. This is needed as the development of nonlinear optical theory in order to get the best quality optical fiber.

## CRediT authorship contribution statement

Harish Abdillah Mardi; Muhammad Ikhwan; Marwan Ramli, Ph.D: Conceived and designed the experiments; Performed the experiments; Analyzed and interpreted the data; Wrote the paper.

Nasaruddin Nasaruddin; Nurmaulidar Nurmaulidar: Analyzed and interpreted the data; Contributed reagents, materials, analysis tools or data; Wrote the paper.

## Declaration of Competing Interest

The authors declare no competing interests.

## Data Availability

No data was used for the research described in the article.

## References

[1] Li M., Xu T., Wang L. (2015). Dynamical behaviors and soliton solutions of a generalized higher-order nonlinear Schrödinger equation in optical fibers. Nonlinear Dyn..

[2] Willner A.E., Khaleghi S., Chitgarha M.R., Yilmaz O.F. (2013). All-optical signal processing. J. Lightwave Technol..

[3] Peng J., Zeng H. (2019). Experimental observations of breathing dissipative soliton explosions. Phys. Rev. Appl..

[4] Peng J., Zeng H. (2018). Build-up of dissipative optical soliton molecules via diverse soliton interactions. Laser Photonics Rev..

[5] Peng J., Sorokina M., Sugavanam S., Tarasov N., Churkin D.V., Turitsyn S.K., Zeng H. (2018). Real-time observation of dissipative soliton formation in nonlinear polarization rotation mode-locked fibre lasers. Commun. Phys..

[6] Biswas A., Zhou Q., Ullah M.Z., Asma M., Moshokoa S.P., Belic M. (2017). Perturbation theory and optical soliton cooling with anti-cubic nonlinearity. Optik.

[7] Yi X., Yang Q.F., Yang K.Y., Vahala K. (2016). Theory and measurement of the soliton self-frequency shift and efficiency in optical microcavities. Opt. Lett..

[8] Song L.M., Yang Z.J., Pang Z.G., Li X.L., Zhang S.M. (2019). Interaction theory of mirror-symmetry soliton pairs in nonlocal nonlinear Schrödinger equation. Appl. Math. Lett..

[9] Arshad M., Seadawy A.R., Lu D. (2017). Modulation stability and optical soliton solutions of nonlinear Schrödinger equation with higher order dispersion and nonlinear terms and its applications. Superlattices Microstruct..

[10] Gao W., Ismael H.F., Husien A.M., Bulut H., Baskonus H.M. (2020). Optical soliton solutions of the cubic-quartic nonlinear Schrödinger and resonant nonlinear Schrödinger equation with the parabolic law. Appl. Sci..

[11] Wang B.H., Lu P.H., Dai C.Q., Chen Y.X. (2020). Vector optical soliton and periodic solutions of a coupled fractional nonlinear Schrödinger equation. Results Phys..

[12] Mendonça J.T., Terças H. (2012).

[13] Gross E.P. (1963). Hydrodynamics of a superfluid condensate. J. Math. Phys..

[14] Fetter A.L. (1966). Vortices in an imperfect Bose gas. IV. Translational velocity. Phys. Rev..

[15] Antoine X., Geuzaine C., Tang Q. (2020). Perfectly matched layer for computing the dynamics of nonlinear Schrödinger equations by pseudospectral methods. Application to rotating Bose-Einstein condensates. Commun. Nonlinear Sci. Numer. Simul..

[16] Liu C., Yu F., Li L. (2019). Non-autonomous wave solutions for the Gross-Pitaevskii (GP) equation with a parabola external potential in Bose-Einstein condensates. Phys. Lett. A.

[17] Kaur P., Roy A., Gautam S. (2021). FORTRESS: FORTRAN programs for solving coupled Gross–Pitaevskii equations for spin–orbit coupled spin-1 Bose–Einstein condensate. Comput. Phys. Commun..

[18] Taniuti T., Washimi H. (1968). Self-trapping and instability of hydromagnetic waves along the magnetic field in a cold plasma. Phys. Rev. Lett..

[19] El-Tantawy S.A., Elgendy A.T., Ismail S. (2017). Cylindrical freak waves in a non-Maxwellian dusty bulk-sheath plasma: an approximate solution for the cylindrical nonlinear Schrödinger equation. Phys. Lett. A.

[20] Sun W.R., Tian B., Liu R.X., Liu D.Y. (2015). Triple Wronskian vector solitons and rogue waves for the coupled nonlinear Schrödinger equations in the inhomogeneous plasma. J. Math. Anal. Appl..

[21] Mabrouk S.M. (2019). Explicit solutions of double-chain DNA dynamical system in (2+1)-dimensions. Int. J. Curr. Eng. Technol..

[22] Ruban V.P. (2020). Discrete vortices on spatially nonuniform two-dimensional electric networks. Phys. Rev. E.

[23] Benjamin T.B., Feir J.E. (1967). The disintegration of wave trains on deep water Part 1. Theory. J. Fluid Mech..

[24] Halfiani V., Fadhiliani D., Mardi H.A., Ramli M. (2018). Nonlinear evolution of Benjamin-Bona-Mahony wave packet due to an instability of a pair of modulations. Int. J. Differ. Equ..

[25] Fadhiliani D., Halfiani V., Ikhwan M., Qausar H., Munzir S., Rizal S., Ramli M. (2020). The dynamics of surface wave propagation based on the Benjamin Bona Mahony equation. Heliyon.

[26] Qausar H., Ramli M., Munzir S., Syafwan M., Susanto H., Halfiani V. (2020). Nontrivial on-site soliton solutions for stationary cubic-quintic discrete nonlinear Schrödinger equation. IAENG Int. J. Appl. Math..

[27] Tchio M.R.S., Abdoulkary S., Mohamadou A. (2019). Modulation instability induced by high-order dispersion to a coupled nonlinear Schrödinger equation in a single-mode optical fiber with Kerr nonlinearity. Phys. Scr..

[28] Agrawal G.P., Haus H.A. (2002). Applications of nonlinear fiber optics. Phys. Today.

[29] Qausar H., Ramli M., Munzir S., Syafwan M., Fadhiliani D. (2021). Soliton solution of stationary discrete nonlinear Schrödinger equation with the cubic-quintic nonlinearity. In IOP Conference Series: Materials Science and Engineering.

[30] Yu W., Zhou Q., Mirzazadeh M., Liu W., Biswas A. (2019). Phase shift, amplification, oscillation and attenuation of solitons in nonlinear optics. J. Adv. Res..

[31] Yin H.M., Tian B., Chai J., Liu L., Sun Y. (2018). Numerical solutions of a variable-coefficient nonlinear Schrödinger equation for an inhomogeneous optical fiber. Comput. Math. Appl..

[32] Lan Z.Z. (2018). Multi-soliton solutions for a (2+1)-dimensional variable-coefficient nonlinear Schrödinger equation. Appl. Math. Lett..

[33] Khater M.M.A. (2021). Diverse solitary and Jacobian solutions in a continually laminated fluid with respect to shear flows through the Ostrovsky equation. Mod. Phys. Lett. B.

[34] Gardner C.S., Greene J.M., Kruskal M.D., Miura R.M. (1967). Method for solving the Korteweg-deVries equation. Phys. Rev. Lett..

[35] Copie F., Randoux S., Suret P. (2020). The physics of the one-dimensional nonlinear Schrödinger equation in fiber optics: rogue waves, modulation instability and self-focusing phenomena. Rev. Phys..

[36] Ablowitz M.J., Musslimani Z.H. (2013). Integrable nonlocal nonlinear Schrödinger equation. Phys. Rev. Lett..

[37] Ma L.Y., Shen S.F., Zhu Z.N. (2017). Soliton solution and gauge equivalence for an integrable nonlocal complex modified Korteweg-de Vries equation. J. Math. Phys..

[38] Wei C.-C., Tian B., Yang D.-Y., Liu S.-H. (2023). Jacobian-elliptic-function and rogue-periodic-wave solutions of a high-order nonlinear Schrödinger equation in an inhomogeneous optical fiber. Chin. J. Phys..

[39] El-Nabulsi R.A., Anukool W. (2023). A family of nonlinear Schrodinger equations and their solitons solutions. Chaos Solitons Fractals.

[40] Wazwaz A.-M. (2022). Bright and dark optical solitons of the (2+1)-dimensional perturbed nonlinear Schrödinger equation in nonlinear optical fibers. Optik.

[41] Stanley U., Olu V.M., Ochonogor C., Amaize P., Francis A. (2018). Experimental analysis of cable distance effect on signal attenuation in single and multimode fiber optics. Int. J. Electr. Comput. Eng..

[42] Makovejs S., Roberts C.C., Palacios F., Matthews H.B., Lewis D.A., Smith D.T. (2015). 2015 Optical Fiber Communications Conference and Exhibition (OFC).

[43] Kashaykin P.F., Tomashuk A.L., Salgansky M.Y., Abramov A.N., Nishchev K.N., Guryanov A.N., Dianov E.M. (2015). Radiation-induced attenuation in silica optical fibers fabricated in high $O_{2}$ excess conditions. J. Lightwave Technol..

[44] Khater M.M.A. (2021). Abundant breather and semi-analytical investigation: on high-frequency waves' dynamics in the relaxation medium. Mod. Phys. Lett. B.

[45] Huang X.B., Xie C., Li H. (2016). Equivalent salt deposit density optical fiber sensor for transmission lines in power grid. IEEE Sens. J..

[46] Song J., Wang J., Niu Y., Wang W., Tong K., Yu H., Yang Y. (2019). Flexible high flux solar simulator based on optical fiber bundles. Sol. Energy.

[47] Al-Buriahi M.S., Alomairy S., Gaikwad D.K., Hegazy H.H., Mutuwong C., Rammah Y.S. (2021). Effects of AgO addition on the mechanical, optical, and radiation attenuation properties of V 2 O 5/P 2 O 5/B 2 O 3 glass system. Appl. Phys. A.

[48] Molina M.I. (2020). The fractional discrete nonlinear Schrödinger equation. Phys. Lett. A.

[49] Al Khawaja U., Al-Marzoug S.M., Bahlouli H. (2017). Peierls–Nabarro potential profile of discrete nonlinear Schrödinger equation. Commun. Nonlinear Sci. Numer. Simul..

[50] Molina M.I. (2018). Solitons in a modified discrete nonlinear Schrödinger equation. Sci. Rep..

[51] Umarov B.A., Ismail N.H.B., Hadi M.S.A., Hassan T.H. (2017). Localized solutions of extended discrete nonlinear Schrödinger equation. J. Phys. Conf. Ser..

[52] Kartono A., Fatmawati V.W., Wahyudi S.T. (2020). Numerical solution of nonlinear Schrödinger approaches using the fourth-order Runge-Kutta method for predicting stock pricing. J. Phys. Conf. Ser..

[53] Cui J., Xu Z., Wang Y., Jiang C. (2021). Mass- and energy-preserving exponential Runge–Kutta methods for the nonlinear Schrödinger equation. Appl. Math. Lett..

[54] Li X., Gong Y., Zhang L. (2020). Two novel classes of linear high-order structure-preserving schemes for the generalized nonlinear Schrödinger equation. Appl. Math. Lett..

[55] Sabirov K.K., Akramov M.E., Otajonov R.Sh., Matrasulov D.U. (2020). Soliton generation in optical fiber networks. Chaos Solitons Fractals.

[56] Mendelson D., Nahmod A.R., Pavlović N., Rosenzweig M., Staffilani G. (2020). A rigorous derivation of the Hamiltonian structure for the nonlinear Schrödinger equation. Adv. Math..

[57] Triki H., Zhou Q., Liu W., Biswas A., Moraru L., Yıldırım Y., Alshehri H.M., Belic M.R. (2022). Chirped optical soliton propagation in birefringent fibers modeled by coupled Fokas-Lenells system. Chaos Solitons Fractals.

[58] Brugnano L., Zhang C., Li D. (2018). A class of energy-conserving Hamiltonian boundary value methods for nonlinear Schrödinger equation with wave operator. Commun. Nonlinear Sci. Numer. Simul..

[59] Chen G., Ma S. (2014). Homoclinic solutions of discrete nonlinear Schrödinger equations with asymptotically or super linear terms. Appl. Math. Comput..

[60] Khater M.M.A. (2021). Diverse solitary and Jacobian solutions in a continually laminated fluid with respect to shear flows through the Ostrovsky equation. Mod. Phys. Lett. B.

[61] Arora G., Rani R., Emadifar H. (2022). Numerical solutions of nonlinear Schrodinger equation with applications in optical fiber communication. Optik.

[62] Zhou T.-Y., Tian B. (2022). Auto-Bäcklund transformations, Lax pair, bilinear forms and bright solitons for an extended (3+1)-dimensional nonlinear Schrödinger equation in an optical fiber. Appl. Math. Lett..

[63] Ahmadianfar I., Heidari A.A., Gandomi A.H., Chu X., Chen H. (2021). RUN beyond the metaphor: an efficient optimization algorithm based on Runge Kutta method. Expert Syst. Appl..

